The article "Predicting Target Genes of San-Huang-Chai-Zhu Formula in Treating ANIT-Induced Acute Intrahepatic Cholestasis Rat Model via Bioinformatics Analysis Combined with Experimental Validation" was published in 2021. Journal: Evid Based Complement Alternat Med.

# Predicting Target Genes of San-Huang-Chai-Zhu Formula in Treating ANIT-Induced Acute Intrahepatic Cholestasis Rat Model via Bioinformatics Analysis Combined with Experimental Validation

**DOI:** 10.1155/2021/5320445

**Published:** 2021-09-01

**Authors:** Jiaming Yao, Junbin Yan, Jinting Wu, Jianshun Yu, Beihui He, Xi Chen, Zhiyun Chen

**Affiliations:** ^1^The First Affiliated Hospital of Zhejiang Chinese Medical University, Hangzhou, Zhejiang 310006, China; ^2^Hangzhou Hospital of Traditional Chinese Medicine, Hangzhou, Zhejiang 310007, China

## Abstract

**Background:**

San-Huang-Chai-Zhu formula (SHCZF) has been used to improve cholestasis for many years. This study aims to predict the possible gene targets of SHCZF in treating acute intrahepatic cholestasis (AIC) in rats.

**Materials and Methods:**

Eighteen SD rats were randomly assigned to the normal group, ANIT group, and ANIT + SHCZF group. Alpha-naphthylisothiocyanate (ANIT) was used to induce AIC. Serum biochemical indexes were detected in each group. After treatment, the livers were collected and used to extract RNA. The library was constructed by TruSeq RNA, sequenced by Illumina, and analyzed by various bioinformatics methods. qRT-PCR was used to verify the target genes related to the efficacy of SHCZF.

**Results:**

Serum ALT, AST, ALP, and TBIL were significantly higher in the ANIT group than in the normal group. Serum ALT and AST levels in the ANIT + SHCZF group were substantially lower than those in the ANIT group. A total of 354 intersected genes were screened by expression level correlation and PCA analysis, GO and KEGG pathway enrichment analysis, and WGCNA and STEM analysis. Then, 4 overlapping genes were found by pathway/BP/gene network construction. SHCZF reversed the downregulation of expression of CYP4A1 and HACL1 and the upregulation of expression of DBI and F11R induced by ANIT. In addition, the qRT-PCR result showed that mRNA expression of CYP4A1, HACL1, and F11R genes in the liver was consistent with the prediction result of bioinformatics analysis.

**Conclusion:**

CYP4A1, HACL1, and F11R are genes related to the occurrence of ANIT-induced AIC in rats and may be considered as targets of SHCZF for the treatment of AIC.

## 1. Introduction

Intrahepatic cholestasis is a primary hepatocellular disorder associated with abnormal formation, secretion, and/or excretion of bile that is asymptomatic in the early stage. Its progression is manifested as jaundice, weakness, dark urine color, and skin pruritus. If left untreated, it may cause cirrhosis, portal hypertension, and liver failure [1]. Until now, no diagnostic criteria for intrahepatic cholestasis have been proposed. Recently, Cao et al. [2] studied the prevalence of cholestasis in the 4660 inpatients with chronic liver disease in Shanghai, China, revealing that ALP level higher than 1.5 times of the upper limit of normal value (ULN) and GGT level higher than 3 times of ULN could be used as diagnostic standards for the disease. Besides, the total incidence of cholestasis was 10.26%, while the distribution of the cholestasis incidence according to the type of chronic liver disease was primary sclerosing cholangitis (PSC) (75%), cirrhosis of various causes (47.76%), and primary biliary cholangitis (PBC) (42.86%) followed by liver tumor (35.97%), autoimmune hepatitis (30.77%), drug-induced liver diseases (28.31%), alcoholic hepatitis (16.46%), and viral hepatitis (5.22%) and nonalcoholic fatty liver disease (2.70%).

Currently, the diagnostic standards of intrahepatic cholestasis have not been wholly unified. The clinical and scientific studies are often based on the 2009 EASL guidelines for clinical practice in treating cholestatic liver disease. The necessary biochemical standards for diagnosing intrahepatic cholestasis are serum ALP level 1.5 times higher than the upper limit of normal (ULN) and the serum GGT level 3 times higher than ULN [1]. Generally, high-risk patients are those with elevated serum bilirubin and serum transaminase and symptoms, such as jaundice, pruritus, and asthenia, as well as those with obvious hepatic inflammatory damage, liver fibrosis, or cirrhosis.

There is no standard effective medicine for the clinical treatment of the disease. S-Adenosylmethionine (SAMe) and ursodeoxycholic acid (UDCA) are the most common drugs used to treat intrahepatic cholestasis. SAMe is a class A drug usually sold as an herbal supplement, which is potentially effective in the treatment of intrahepatic cholestasis during pregnancy. Nonetheless, SAMe has not yet been approved by the Food and Drug Administration (FDA). Jiang et al. [3] searched the cases of adverse drug reaction (ADR) caused by SAMe reported in databases up to 2017 and found that increase in the application led to many reports on Adverse drug reaction (ADR) related to multiple human systems, some of which have not been recorded in the medicine instructions. On the other hand, UDCA is a first-line drug approved by the FDA to treat primary biliary cirrhosis (PBC)/primary biliary cholangitis (PBC). It has high safety and tolerance, but many patients have no response [4]. Glucocorticoid is another drug used in patients with cholestasis mediated by immune mechanism; however, the treatment benefits and possible adverse reactions should be carefully considered before use. Moreover, the FDA has recently approved obeticholic acid for patients with cholestasis [5], but the clinical effectiveness and safety of the drug still need to be evaluated via future trials. Also, other medicines, which are currently being researched, or are in the developmental stage, include fenofibrate and norUDCA [6–9].

The exact pathogenesis of intrahepatic cholestasis has not yet been fully elucidated, which affects the development of therapeutic drugs. It is believed that the pathogenesis of intrahepatic cholestasis is mainly related to genetic defects, expression changes or dysfunction of bile acid transporters [10, 11], oxidative stress in the liver [12], and changes in intestinal flora [13]. Currently, the molecular target study on drug therapy mainly focuses on exploring nuclear receptors. The nuclear receptor ligands include endogenous and exogenous molecules, such as hormones, fatty acids (FA), bile acids (BA), drugs, toxins, and metabolic intermediates. It has been discovered that nuclear receptors (NR) such as farnesoid *X* receptor (FXR), liver *X* receptor (LXR), pregnane *X* receptor (PXR), peroxisome proliferator-activated receptor (PPAR-*α*/*γ*/*δ*), and small heterodimer partner (SHP) can regulate bile acid homeostasis, bile synthesis and secretion, liver inflammation, regeneration, fibrosis, and tumor formation through ligands [14–16]. Other potential targets include G-protein coupled receptor 5 (TGR5) [17, 18], ASBT inhibitor [7], and miRNAs [19].

So far, several animal models for studying intrahepatic cholestasis have been developed, including the ANIT induction model, lipopolysaccharide induction model, estradiol estrogen benzoate induction model, chlorpromazine induction model, rifampin induction model, cholic acid induction model, and 3,5-diethoxycarbonyl-1,4-dihydrocollidine (DDC) model. Alpha-naphthyl isothiocyanate (ANIT) is a common hepatotoxicant experimentally used to reproduce the pathologies of drug-induced liver injury of the bile duct, which in turn causes an elevation in ALP, GGT, TBIL, ALT, and AST levels. Its biochemical and pathological changes are similar to those of human intrahepatic cholestasis [20].

Jaundice is the main symptom of acute intrahepatic cholestasis (AIC). In China, traditional Chinese medicine has been used to treat jaundice for at least 2000 years. San-Huang-Chai-Zhu formula (SHCZF) is an improved medicine based on the Da-Huang-Xiao-Shi formula (standard prescription; a mix of herbs that have been used for the treatment of jaundice for many years). SHCZF is composed of 5 traditional Chinese medicines: *Rheum officinale Baill.* (Da Huang, DH), *Phellodendron chinense Schneid.* (Huang Bai, HB), *Gardenia jasminoides Ellis.* (Zhi Zi, ZZ), *Bupleurum chinensis DC.* (Chai Hu, CH), and *Atractylodes macrocephala Koidz.* (Bai Zhu, BZ). Zhang et al. have confirmed that *Rheum officinale Baill.*, monarch drug (drugs that play the major role in the formula) in SHCZF, could treat cholestasis rats by improving bile acid metabolism [21]. In addition, our previous study has directly identified SHCZF has a good effect in treating acute intrahepatic cholestasis [22].

Traditional Chinese medicine (TCM) compounds are a relatively complex system due to their multiple drug components, synergistic effects, and multiple therapeutic targets. This is precisely the advantage of TCM, but it will also cause problems such as difficulty in clarifying the therapeutic targets, which is not conducive to elucidating the therapeutic mechanism and clinical promotion of TCM. Therefore, we tried to screen clear targets of SHCZF in the treatment of cholestasis through sequencing technology combined with bioinformatics analysis and experimental verification to provide theoretical support for the promotion and further in-depth study of SHCZF.

## 2. Materials and Methods

### 2.1. SHCZF Component Analysis

SHCZF is composed of rhubarb, phellodendron, gardenia, bupleurum, and atractylodes macrocephala (Table 1). SHCZF is composed of rhubarb, phellodendron, gardenia, bupleurum, and atractylodes macrocephala in the ratio of 4 : 4 : 3 : 3 : 4. Add 10 times the amount of water to the abovementioned herbal medicine, soak for 30 minutes, and boil for 1.5 hours; filter out the liquid; add 8 times the amount of water to the medicinal residue, and decoct for 1 hour after boiling; filter out the liquid; add 6 times the amount of water, and decoct for 0.5 hours after boiling. Finally, combine the three decoctions and concentrate into the extract (2 g/ml). The above extract was processed by the pharmaceutical center of The First Affiliated Hospital of Zhejiang Chinese Medical University. The representative components of the formula were determined by high-performance liquid chromatography (HPLC). The following analytical conditions were used: liquid phase: Shimadzu LC-20AT HPLC; chromatographic column: Agilent Extend-C18 (250 mm × 4.6 mm, 5 *μ*m); mobile phase A: 0.1% phosphoric acid, B: acetonitrile; gradient elution: 0–10.00 (min) pump A: 90%; B. conc 10%; 10–20.00 (min) pump A: 30% B. conc 30%; 20–30.00 (min) pump A: 40% B. conc 60%; 30–45.00 (min) pump A: 30%; B. conc 70%; 45–53.00 (min) pump A: 30%; B. conc 70%; 53–54.00 (min) pump A: 90%; B. conc 10%; 59.00 min controller stop. According to the comparison of standards and calculation by one-point external standard method, the content of aloe-emodin was 0.030863 mg/g, chrysophanol was 0.024877 mg/g, rhein was 0.099097 mg/g, emodin was 0.022389 mg/g, emodin methyl ether was 0.006596 mg/g, berberine was 1.362123 mg/g, and the gardenoside was 3.993566 mg/g based on external standard (Figure 1).

### 2.2. Experimental Animals and Treatment

Eighteen male SD rats (SPF grade) weighing 130–150 g were provided by Shanghai SIPPR-Bk Laboratory Animal Co., Ltd. All the animals were housed in an environment with a temperature of 20–24°C, relative humidity of 60 ± 5%, a light/dark cycle of 12/12 hr, and allowed food and water ad libitum. All animal studies (including the mice euthanasia procedure) were done in compliance with the regulations and guidelines of Zhejiang Chinese Medical University institutional animal care and conducted according to the AAALAC and the IACUC guidelines (no. SCXK (Shanghai) 2013–0016 and animal ethics no. ZSLL-2015-79).

After one week of acclimation, animals were randomly divided into the normal, ANIT, and ANIT + SHCZF groups (six animals in each group). On the first day, rats in the ANIT + SHCZF group received 20 g/kg SHCZF (the dosage of SHCZF is obtained by equivalent conversion based on the best dose of clinical medication) once a day for 5 days by gavage, while rats in the normal and ANIT groups were given the same volume of 0.9% NaCl every day for 5 days. On the third day, the rats in the normal group received 1 ml/kg sesame oil, while the other two groups were given 4% ANIT (provided by J&K Scientific, Lot no. 249447) 100 mg/kg (the dosage of ANTI referred to in the literature [23, 24]) that was prepared in sesame oil. The rats in each group were treated after 48 h of ANIT or sesame oil administration, respectively. The rats fasted for 16 h before the sacrifice (5 PM to 9 AM at the next day).

### 2.3. Blood and Liver Collection

Blood was collected from the abdominal vein after anesthesia with 3% pentobarbital sodium in the morning of the same day. Serum was separated, and TBIL, ALT, AST, and ALP levels were detected by automatic biochemical instrument (the kits were provided by Shanghai Senneng Desai Diagnostic Technology Co., Ltd., Lot no. 14108170201, 14127070201, 14126070201, and 14104170202, respectively).

Besides, after the treatment was completed, the liver was collected and snap-frozen in liquid nitrogen and then reversed at −76°C for 3 h.

### 2.4. High-Throughput Whole Gene Transcriptome Sequencing

The livers from three rats were selected from each group. Total RNA was extracted by TRIzol reagent (Invitrogen, USA). The purity and concentration of total RNA were analyzed by Agilent 2100 biological analyzer and RNA 6000 Nano LabChip Kit (Agilent, USA), and the RIN value was >7. Qualified RNA samples were amplified to construct a library. Three groups of samples were sequenced by Illumina high-throughput sequencing, which was completed by Shanghai Yuanzi Biotechnology Co., Ltd., of China, as shown in Figure 2.

### 2.5. Data Analysis

#### 2.5.1. Quality Control of Sequencing Data

Raw sequence data (raw reads) obtained by sequencing might contain unqualified sequence data, such as low overall quality and low-end quality, which could be used for data analysis using Trimmomatic (v3.6) [25] (http://www.usadellab.org/cms/index.php?page=trimmomatic). We used the following steps to control the quality of original offline data: (A) removing the bases whose continuous mass was <10 at both ends of the reads; (B) removing the bases whose mass was <80% and >20; and (C) filtering out reads with length <50 nt. Then, TopHat2 software (V 2.1.0) [26] (http://ccb.jhu.edu/software/tophat/index.shtml) was used to locate clean reads to the GENCODE database (https://www.gencodegens.org/releases/current.html) rat reference genome (RNO6.0, Ensembl) [27]. At most, four base mismatches were allowed, and default parameters were used for the rest. StringTie tool (v1.3.3b) was used (http://ccb.jhu.edu/software/stringtie/index.shtml) [28] to reassemble the transcripts of nine samples, respectively, and fuse the generated GTF files into a more comprehensive transcript annotation result. HTSeq (v0.9.1) tool (https://htseq.readthedocs.io/en/release_.9.1) [29] and Cuffquant and Cuffnorm of Cufflinks (v2.2.1) [30] (http://cole-trapnell-lab.github.io/cufflinks/) were then used to quantitatively analyze the expression level of genes and transcripts in a single sample.

#### 2.5.2. Distribution and Comparative Analysis of Expression Abundance between Samples

The correlation of expression levels between samples is an important index to test the reliability of experiments and the rationality of sample selection. Therefore, based on the expression abundance of each sample, varieties of methods were used to evaluate the correlation between samples: (1) Cor function (https://stat.ethz.ch/R-manual/R-devel/library/stats/html/cor.html) in R3.4.1 was used to calculate the Pearson correlation coefficient between each pair of samples. The closer the correlation coefficient was to 1, the higher the similarity of expression patterns between samples was. (2) Using psych package (version 1.7.8) in R3.4.1 (https://cran.r-project.org/web/packages/psych/index.html), all samples were analyzed by principal components analysis (PCA) based on expression abundance.

#### 2.5.3. Screening of Significant Difference in Gene Expression Levels between Groups

The normal group (group A), the ANIT group (group B), and the ANIT + SHCZF treating group (Group C) were divided into two comparison groups: group B versus A that was used to investigate disease-related genes, and group C versus B to examine crucial genes and mechanism of SHCZF treatment. Limma package [31] (version 3.32.5) (http://bioconductor.org/packages/release/bioc/html/limma.html) in R3.4.1 was then used to screen the significantly different expression genes from the two comparison groups. FDR value <0.05 and |logFC| > 1 were used as the threshold value of the significantly different expression genes. For the obtained genes, pheatmap package version 1.0.8 [32] (https://cran.r-project.org/web/packages/pheatmap/index.html) in R3.4.1 was used to cluster the expression values of the samples based on the “correlation” algorithm. Afterward, David 6.8 [33, 34] (https://david.ncifcrf.gov/) online search software was used to enrich GO function and KEGG pathway of genes with significant variation in expression levels (significant correlation threshold: FDR less than 0.05).

#### 2.5.4. Further Screening of Disease-Related Genes

Union of the two groups of significantly differentially expressed genes screened in the previous step was taken, and the set of genes was further analyzed:

  (1) Screening of genes associated with different status weighted gene coexpression network analysis (WGCNA) package [35] (version 1.61) (https://cran.r-project.org/web/packages/WGCNA/) in R3.4.1 was used to analyze and screen the union of genes, and the gene modules significantly related to different status (normal/disease/drug administration) were obtained.
  (2) Cluster analysis of gene expression in different status for gene expression profile data in different status (normal/disease/drug administration), STEM [36] (short time-series expression miner) (version 1.3.11) (http://www.cs.cmu.edu/∼jernst/stem/) software was used to cluster genes with significantly similar expression patterns with the status change (threshold: correlation between gene expression in the same class was higher than 0.8, and *p* value <0.05).

The essential genes screened by (1) and (2) were intersected; the genes with significantly similar expression changes in different statuses and especially related to various disease states were obtained for further analysis.

#### 2.5.5. Construction of Disease-Related Pathway/BP/Gene Network

For the intersection gene set with significant similarity obtained in the previous step, the biological process of GO and enrichment analysis of the KEGG pathway were performed by David 6.8. The pathway/BP/gene regulatory network was constructed for the biological processes, KEGG pathways related to gene enrichment, and the differentially expressed genes involved.

“Cholestasis” was used as the keyword in Comparative Toxicogenomics Database (http://ctd.mdibl.org/) [35] to search for the KEGG pathway and genes directly related to cholestasis and map to the gene pathway/BP/gene network constructed, through which the essential genes involved in different biological processes and disease pathways were observed. Network visualization was carried out by Cytoscape 3.6.0 (http://www.cytoscape.org/) [36].

### 2.6. Fluorescence Quantitative PCR Validation

Six rats from each group were selected to extract total RNA using the Extraction Kit (Takara MiniBEST universal RNA extraction kit, TAKARA) from the liver. The purity and content of total RNA were measured using Nanodrop micro nucleic acid analyzer. The extracted total RNA was synthesized into cDNA using a PrimeScript™ RT Master Mix (Perfect Real Time, TAKARA) and amplified using a qPCR kit (SYBR® Premix Ex Taq™ II, Tli RNaseH Plus, TAKARA) using cDNA as a template. Primers were designed and synthesized by Sangon (Table 2). *β*-Actin was used as an internal reference gene. The mRNA expression of each gene in the liver was calculated by 2^−ΔΔ*CT*^.

### 2.7. Statistical Analysis

SPSS21.0 was used to analyze the data of serum liver function and fluorescence quantitative PCR, which were expressed as mean ± standard deviation. All data were transformed into normal distribution after normal tests. Single-factor analysis of variance was used. LSD method was used to compare the homogeneity of variance. Dunnett's T3 method was used to compare the homogeneity of variance. *p* < 0.05 was considered to be statistically significant.

## 3. Results

### 3.1. Effect of SHCZF on Serum Liver Function in Intrahepatic Cholestasis Rats

Our data indicated that serum levels of ALT, AST, ALP, and TBIL in the ANIT group were significantly higher than those in the normal group (*p* < 0.01). The serum levels of ALT and AST in the ANIT + SHCZF group were significantly lower compared to the ANIT group (*p* < 0.01), while there was no significant difference in ALP and TBIL levels (*p* > 0.05) (Figure 3). These findings suggested that SHCZF has a significant protective effect on AIC.

### 3.2. Quality Control of Gene Sequencing Data

A total of 233,577,888 original sequences were obtained by high-throughput transcription sequencing from 9 samples, with an average base sequencing error rate of 0.02%. After filtering out the unqualified low-quality data (including those with joints and low-quality data), 231,585,315 high-quality sequences (clean reads) were obtained, accounting for 99.15% of the total. Then, using TopHat software algorithm, clean reads were compared to the reference genome; the results showed that the sequences that could be compared to the genome accounted for 85.97% of the total clean reads, 77.93% of which had unique location. Next, FPKM expression value of each sample was obtained through Cufflinks software. The correlation between samples was evaluated by various methods based on the expression abundance of each sample: (1) calculating Pearson's correlation coefficient between every two samples (Figure 4(a)); the square distribution of the correlation coefficient *R* between samples was 0.6–1, and the average sample correlation was 0.806. (2) The results of PCA analysis based on expression abundance of samples (Figure 4(b)); overall, all samples were relatively clustered, indicating that the individual differences of samples in the same group were not too significant. Samples in the same group tended to be distributed in the same area, thus suggesting that the differences between samples in the same group were insignificant. Therefore, the integrity of the samples was almost ideal, and there were no scattered samples.

### 3.3. Screening of Significant Differences in Gene Expression Levels between Groups

A total of 960 (467 downregulated and 493 upregulated) and 423 (208 downregulated and 215 upregulated) differentially expressed genes meeting the threshold were screened after comparing the normal group (group A), the ANIT group (group B), and the ANIT + SHCZF group (group C). Bidirectional hierarchical clustering was conducted based on the significantly differentially expressed genes screened from the two groups. As shown in Figure 5, the difference of the genes screened in the two groups between samples of different types was significant with sample characteristics.

Next, GO enrichment and KEGG pathway enrichment analysis were performed on significantly differentially expressed genes in the ANIT group versus the normal group and the ANIT + SHCZF group versus the ANIT group. Twenty-seven GO functions (11 BP, 8 CC, and 8 MF) and 26 GO functions (13 BP, 7 CC, and 6 MF) with significant correlations were obtained, as shown in Figure 6. The differentially expressed genes in the ANIT + SHCZF group and the ANIT group were significantly related to the biological process of steroid and cholesterol metabolism. From the results of pathway enrichment, the differentially expressed genes in the two groups were related to fatty acid metabolism, steroid synthesis, PPAR signal pathway, etc.

### 3.4. Screening of Disease Status-Related Genes

To further screen the genes related to the disease, the significant differential expression gene sets in group B versus group A and group C versus group B were compared. As shown in Figure 7, the two sets of genes were merged, and a total of 1177 genes were selected for analysis in the next step.

#### 3.4.1. WGCNA Analysis

Weighted correlation network analysis (WGCNA) was used to screen the gene sets with highly synergistic changes in expression. The potential targets for SHCZF treatment of cholestasis were selected according to the association between the connectivity of above 1177 differentially expressed genes and the disease state.

To meet the premise of scale-free network distribution, the value of the weight parameter power of the adjacency matrix was analyzed. The selection range of network construction parameters was set, and the scale-free distribution topology matrix was calculated. As shown in Figure 8(a), the value of power was selected when the square value of the correlation coefficient reached 0.9 for the first time, that is, power = 16. Under this coefficient, the weight constructed jointly represented that the average connectivity of nodes in the network was 1, which satisfied the connectivity property of nodes in the scale-free network. Then, the dissimilarity coefficient between genes was calculated to get a system-clustering tree. According to the hybrid dynamic cutting tree standard, the minimum number of genes in each gene module was set as 50, and the pruning height as cutHeight = 0.99. As shown in Figure 8(b), 8 related modules were screened. Finally, the correlation between each module and the different disease statuses (normal/disease/administration) was calculated. The significant correlation *p* value between the whole module and different disease statuses was 0.0019 (Figure 8(c)). Among the eight modules, four (black, yellow, red, and turquoise) were positively correlated with disease status, and the correlation coefficient was higher than 0.8. Therefore, the genes contained in these four modules (a total of 499 genes) were positively correlated with disease status.

#### 3.4.2. STEM Analysis

STEM software was used to analyze the expression of above 1177 differentially expressed genes, and gene clusters with similar expression patterns were screened. Four classes were obtained with gene expression similarities higher than 0.8 and *p* < 0.05 as screening thresholds. The expression patterns in each cluster set varied with the status (Figure 9). The pattern of red class indicates that the gene expression was downregulated in the ANTI group and upregulated after the treatment of SHCZF. In the green and blue classes, the expression of genes in the group was first upregulated and then decreased after treatment. In the yellow class, most of the genes were continuously increased, and a few of the genes were firstly increased in the ANTI group and then slightly downregulated after SHCZF treatment. Each class contained 370, 204, 170, and 69 genes, respectively.

A comprehensive comparison was made between the 499 genes that significantly correlated with disease status in (1) and the 813 gene sets in the 4 classes (color markers) clustered considerably with the status change in (2), as shown in Figure 10. The two gene sets shared 354 intersected genes. This part of the intersected genes was taken as the genes related to cholestasis progression and SHCZF treatment and subject for further analysis.

### 3.5. Enrichment Analysis of KEGG and GO

First, enrichment analysis of GO biological process and KEGG pathway for 354 intersected genes screened was conducted. As shown in Figure 11 and Table 3, 13 significantly related GO biological processes (all BP, not enriched to MF and CC) and 9 pathways were obtained. The results showed that the shared genes were significantly related to the biological processes, such as immune response, fatty acid metabolism, PPAR signaling pathway, and fatty acid metabolism.

### 3.6. Construction of Disease-Related Pathway/BP/Gene Network and Screening of Potentially Therapeutic Genes

We synthesized biological processes and pathways involved in 354 intersection genes to construct pathway/BP/gene networks related to cholestasis, as shown in Figure 12. There are 150 gene nodes (14 BPs, 9 pathways, and 127 gene nodes) and 377 connecting edges.

A total of 172 KEGG pathways and 9 genes directly related to cholestasis were found in the CTD database using “cholestasis” as the keyword.

Firstly, the pathways found in CTD were mapped to the pathway/BP/gene network. A total of six diseases related pathways overlap KEGG pathways (pathways marked with ^*∗*^ in Table 3, a bright blue square node in Figure 12), which were seen as SFCZF treating pathway of cholestasis mice (involved 41 unique genes). The 6 intersection pathways are, respectively, the PPAR signaling pathway (rno03320), fatty acid metabolism (rno00071), retinol metabolism (rno00830), antigen processing and presentation (rno04612), cell adhesion molecule (CAMs) signaling pathway (rno04514), and leukocyte cross endothelium migration pathway (rno04670).

Based on the expression level of the 41 unique genes mentioned above, combined with the results of STEM analysis, we further screened genes that may be related to both disease occurrence and pharmacodynamic response according to the expression changing trend. CYP4A1 and ADH7 in class 1 were downregulated in the ANIT group compared with that in the normal group (B vs. A). The expression of the above two genes in the SHCZF + ANIT group was upregulated compared with the ANIT group (C vs. B). The expression of ACTG1, CD74, DBI, F11R, ITGB1, PVR, RFX5, RT1-N2, RT1-N3, RT1-S3, and SDC4 in class 3 was significantly upregulated in the ANIT group compared with that in the normal group (B vs. A). The expression of these eleven genes was significantly downregulated in the SHCZF + ANIT group compared with that in the ANIT group (C vs. B).

Subsequently, the screened 9 cholestasis-related disease genes were mapped into the disease-related pathway/BP/gene network (Figure 12). There were four overlapping genes: NQO1, ABCC3, NFE2L2, and HACL1. NQO1 is involved in the redox biological process, ABCC3 in the stimulation response, NFE2L2 in the organic response process, and HACL1 in the fatty acid metabolism process. Furthermore, genes related to both disease progression and pharmacodynamic response were screened according to the trend of expression changes (selected genes were required to be a disease gene whose expression had changed significantly before and after treatment). Among the above 4 genes, only HACL1 was significantly downregulated in group B versus A and upregulated in group C versus B, suggesting that the changes in the expression level of HACL1 might be related to both disease occurrence and SHCZF treating response.

Therefore, we preliminarily screened the following 14 genes that might be related to the occurrence of disease and the response of drug efficacy according to their changing characteristics. The expression of CYP4A1, ADH7, and HACL1 was downregulated in group B versus A. The expression of these three genes was upregulated in group C versus B. The expressions of ACTG1, CD74, DBI, F11R, ITGB1, PVR, RFX5, RT1-N2, RT1-N3, RT1-S3, and SDC4 were all upregulated in group B versus A. The expression of these eleven genes was downregulated in group C versus B. Combined with the current studies on the functions of the above genes, we further screened the genes involved in the regulation of liver inflammation and bile acid metabolism and obtained four genes: CYP4A1, DBI, HACL1, and F11R (Figure 13).

### 3.7. Expression of CYP4A1, DBI, HACL1, and F11 R mRNA Detected by qRT-PCR

The expression of CYP4A1 and HACL1 mRNA in the liver was downregulated in the ANIT group compared with that in the normal group (*p* < 0.01), while the expression of CYP4A1 and HACL1 mRNA was upregulated in the SHCZF + ANTI group compared with that in the ANIT group (*p* < 0.05 and *p* < 0.01). The expression of F11R mRNA was upregulated in the ANIT group compared with that in the normal group (*p* < 0.01), while the expression of F11R mRNA was downregulated in the SHCZF + ANIT group compared with that in the ANIT group (*p* < 0.01). DBI mRNA expression in the ANIT group was significantly downregulated compared with that in the normal group, and no statistical difference was found between the SHCZF + ANIT group and the ANIT group (*p* > 0.05) (Figure 14). The expression change of DPI verified by qRT-PCR was inconsistent with the sequencing results. We think this may be due to the different sample sizes. We only selected 3 rats from each group for sequencing, but 6 rats from each group were selected for qRT-PCR validation. A small sample size for sequencing may cause occasional errors. The results showed that SHCZF could significantly improve the expression of CYP4A1, HACL1, and F11R mRNA, but could not significantly improve the expression of DBI mRNA.

## 4. Discussion

The sequencing data indicated that SHCZF possesses a preventive and therapeutic effect on the ANIT-induced AIC rat model. Four possible pharmacodynamics gene targets of SHCZF, CYP4A1, DBI, HACL1, and F11R were screened by bioinformatics analysis. Subsequently, the validation of fluorescent quantitative PCR was performed, indicating that the mRNA expression of CYP4A1, HACL1, and F11R was consistent with the predictive results.

CYP4A1 and DBI are involved in the PPAR signaling pathway, which is related to cholestasis. PPAR-*α* mediates the development of cholestasis and has an essential role in maintaining the homeostasis of bile acid metabolism [37, 38]. In a previous study, wild-type and PPAR-*α*-null mice were treated with cholic acid (CA) to evaluate the role of PPAR-*α* in bile acid homeostasis [38]. After the intervention, the PPAR-*α*-null mice showed an accumulation of intrahepatic bile acid, which was not observed in wild-type mice. The CYP4A1 gene of rats corresponds to CYP4A11 in mice and the human body, which belongs to CYP450 I-phase metabolizing enzyme. The latter is widely involved in the metabolism of exogenous substances, such as various drugs, prepoisons, and precarcinogens, as well as the metabolism of endogenous substances, such as bile acid, steroid hormone, and arachidonic acid. Over the recent years, it has been found that PPAR-*α* is widely involved in regulating P450 metabolizing enzymes; CYP4A1 is its downstream target gene, which is widely used for the determination of PPAR-*α* activation [39]. In this study, the result of liver gene sequencing and qRT-PCR suggested that CYP4A1 was downregulated in the occurrence of ANIT-induced AIC and upregulated in the SHCZF group, thus suggesting that CYP4A1 has a vital role in the occurrence of AIC. This data also indicated that CYP4A1 might be a vital gene target for SHCZF to prevent and treat AIC.

Diazepam binding inhibitor (DBI), also known as acetyl-CoA binding protein (ACBP) or cholecystokinin releasing peptide (CCK-RP), is a hormone-regulated protein, which is mainly expressed in the liver, brain, and testis. It can regulate lipid metabolism and other biological processes [40]. DBI regulates the biosynthesis of steroids and bile acids through peripheral benzodiazepine receptors [41]. The overexpression of DBI in the liver downregulates the expression of PPARs, and DBI itself is the target gene of PPAR [42]. In this study, the result of liver gene sequencing suggested that DBI was upregulated in the occurrence of ANIT-induced AIC and down-regulated in the SHCZF group. Nevertheless, the subsequent qRT-PCR results indicated that DBI was downregulated in the occurrence of ANIT-induced AIC, and there was no significant difference between the SHCZF group and the ANIT group. The results of the above two detection methods were inconsistent and thus need to be further investigated in the future.

2-Hydroxyacyl-coA lyase (HACL1) is a critical enzyme in the *α*-oxidation process of phytate oxidase discovered in 1999. Previously, HACL1 was considered to have an essential role in the degradation of 3-methyl branched fatty acids (such as phytic acid) and the shortening of 2-hydroxy long-chain fatty acids. Recently [43], it has been found that under normal conditions, mice lacking HACL1 do not show specific phenotypes. However, after adding chlorophyllin in the feed, phytic acid accumulates in the tissues, mainly in the liver and serum of mice. Due to the toxic effect of phytic acid (or metabolite), the animal weight was significantly reduced, and there was no white adipose tissue in the abdomen. The liver was swollen and mottled, and glycogen and triglyceride in the liver were also reduced. Moreover, PPAR-*α* in the liver was activated. The above results suggest that HACL1 might be related to PPAR-activation in the liver; however, the exact mechanism of action needs to be further explored. In this study, the results of gene sequencing and qRT-PCR of the liver suggested that the expression of HACL1 was downregulated in the ANIT-induced AIC and upregulated in the SHCZF group. We speculate that HACL1 may be involved in cholestasis through the PPAR-*α* related signaling pathway, and it may be the gene target of SHCZF.

F11R, also known as junctional adhesion molecule A (JAM-A), or JAM-1 and JAM1, is a crucial membrane protein that forms tight junctions. It appears in the early stage of tight junction establishment and is enriched in the tight connections between epithelial cells with proteins such as occludin and claudin. It is expressed in the liver, the intestine, and other tissues, and it regulates cell proliferation, tumor invasion and metastasis, and intestinal mucosal barrier dysfunction. Previous studies have reported enhanced intestinal epithelial permeability, bacterial translocation, and increased colonic lymphocytes in mice models lacking F11R [44]. F11R is a new candidate gene related to microscopic colitis (MC) [45]. Recently, it has been discovered that F11R is related to some liver diseases. After feeding with high saturated fat, fructose, and cholesterol, F11R (−/−) in treated mice was characterized by severe steatohepatitis compared to the control ones [46]. Moreover, the lower level of JAM-A was found in the colon mucosa of NAFLD patients compared to healthy individuals. The lower expression of JAM-A is related to the higher level of inflammation in the colon mucosa [46]. The metabolism of bile acid is easily affected by the changes in intestinal structure and function due to enterohepatic circulation. The determination of the critical regulatory mechanism of enterohepatic circulation can be used as a drug target for cholestatic liver disease [47]. In this study, the results of gene sequencing and qRT-PCR of liver tissue suggested that F11R expression was upregulated in ANIT-induced AIC and downregulated in the SHCZF group compared with the former. We presume that the expression of F11R in the liver has an essential role in ANIT-induced AIC, which may be the significant gene target for the prevention and treatment of AIC by SHCZF. However, the specific mechanism of the gene target needs to be further examined.

As a preliminary exploration of the ANIT-induced AIC rat models and the pharmacodynamics gene target of SHCZF, the study identified the target of SHCZF for the treatment of cholestasis in rats. However, there is a lack of in-depth research on the overall pathway or mechanism, which needs to be improved in future work. In addition, in the future, gene knockout mice and different types of cholestasis animal models should be established to further investigate the pharmacodynamic mechanism of those genes.

## 5. Conclusion

In this study, we investigated the effect of SHCZF on the prevention and treatment of ANIT-induced AIC in rats. By sequencing and bioinformatics analysis, CYP4A1, HACL1, F11R, and DBI were identified as possible pharmacodynamic gene targets of SHCZF in treating cholestasis rats. Through qRT-PCR, CYP4A1, HACL1, and F11R were finally confirmed as the therapeutic targets of SHCZF.

## Figures and Tables

**Figure 1:** Representative chromatogram of significant compounds in SHCZF. (a) 1: aloe emodin; 2: emodin; 3: rhubarb acid; 4: chrysophanol; and 5: emodin methyl ether. (b) 6: berberine. (c) 7: gardenoside.

**Figure 2:** Sequencing analysis of Illumina.

**Figure 3:** Changes in serum ALT, AST, ALP, and TBIL in different rat groups ($\bar{x}\pm s$, IU/L, *n* = 6). Compared with normal group ^*∗∗*^*p* < 0.01; compared with ANIT group ^ΔΔ^*p* < 0.01.

**Figure 4:** (a) Pairwise correlation heat maps of samples based on expression abundance. The changes in color from a light color to dark color represent the relationship of the correlation coefficient between samples from small to large. The horizontal and vertical axes represent the names of samples, and the numbers in each grid represent the correlation coefficient. (b) PCA diagram of samples based on expression abundance. *x-*, *y-*, and *z-*axes represent PC1, PC2, and PC3, respectively. Black circle, red square, and green triangle represent the samples of groups A, B, and C, respectively.

**Figure 5:** (a) Volcanic map (left) and two-way tomographic cluster map (right) of genes with significantly different expression in group B versus group A. (b) Volcanic map (left) and two-way tomographic cluster map (right) of genes with significantly different expression in group C versus group B.

**Figure 6:** (a) GO function annotation and KEGG pathway significantly related to differential gene in group A versus B. (b) GO function annotation and KEGG pathway significantly related to differential gene in group B versus C. Red, black, green, and blue squares represent KEGG, MF, CC, and BP, respectively. Size of the squares represents −log_2_ (FDR).

**Figure 7:** Venn diagram of significant differential expression gene sets in group B versus A and group C versus B.

**Figure 8:** (a) Power selection diagram of adjacency matrix weight parameters (left). The horizontal axis represents weight parameter power, and the vertical axis represents a square of the correlation coefficient between log (*k*) and log (*p* (*k*)) in the corresponding network. The higher the square value of the correlation coefficient is, the closer the network is to the distribution without the network scale. The red line indicates the standard line where the square value of the correlation coefficient reaches 0.9. (Right) Schematic diagram of the average connectivity of gene nodes in the coexpression network constructed under different power parameters. The red line shows the average connectivity of network nodes (1) under the power parameter of the adjacency matrix on the left. (b) Module division tree diagram. Each color represents a different module. (c) The modular histogram shows a significant correlation between disease statuses. Each color represents a different module.

**Figure 9:** Cluster analysis of gene expression profile. Each small square represents the different clustering gene class obtained by stem. The black line in the square indicates the overall trend of expression of all genes in the gene set; the number in the lower left represents the significant *p* value of the similarity of gene expression in the cluster.

**Figure 10:** Comparison of STEM and WGCNA gene sets.

**Figure 11:** GO biological process and KEGG pathway histogram were correlated with the shared genes. The horizontal axis represents the number of genes; the vertical axis represents the name of the biological process and KEGG pathway; and column colors from green to red represent the significance from low to high.

**Figure 12:** Pathway/BP/gene network map related to cholestasis disease. Red, green, purple, and yellow round points, respectively, represent genes in the class 1–4 set with significantly similar expression in STEM. Blue square points represent pathways (bright blue points represent pathways related to cholestasis diseases recorded in the CTD database), and blue diamond points represent biological processes. Each “P” and “B” correspond to the names in the table below the network.

**Figure 13:** CYP4A1, DBI, HACL1, and F11R genes expression in the liver. CYP4A1 and HACL1 were downregulated in group B versus A and upregulated in group C versus B. DBI and F11R were upregulated in group B versus A and downregulated in group C versus B. (a) CYP4A1, (b) DBI, (c) HACL1, and (d) F11R.

**Figure 14:** mRNA expression of CYP4A1, DBI, HACL1, and F11R detected by qRT-PCR (mean ± standard deviation, *n* = 6). Compared with the normal group ^*∗∗*^*p* < 0.01; compared with the ANIT group ^Δ^*p* < 0.05 and ^ΔΔ^*p* < 0.01.

**Table 1:** The compositions of SHCZF.

Chinese name	Family	Latin name	Parts used	Proportion
Da Huang, DH	Polygonaceae	*Rheum officinale* Baill.	Rhizoma	22.22%
Huang Bai, HB	Rutaceae	*Phellodendron chinense* Schneid.	Bark	22.22%
Zhi Zi, ZZ	Rubiaceae	*Gardenia jasminoides* Ellis.	Fruit	16.67%
Chai Hu, CH	Apiaceae	*Bupleurum chinensis* DC.	Root	16.67%
Bai Zhu, BZ	Compositae	*Atractylodes macrocephala* Koidz.	Rhizoma	22.22%

**Table 2:** Fluorescence quantitative PCR primers.

Rat CYP4A1		
Upstream primer	Sense	AATGGCAGTGTTCAGGTGGATGG
Downstream primer	Antisense	GGCAAGTTGACAAGCACGGTTG

Rat HACL1		
Upstream primer	Sense	CATGTTCGGTGTCGTAGGCATCC
Downstream primer	Antisense	GCCGCTTGCTCATTCCTCATCC

Rat DBI		
Upstream primer	Sense	CGCCTCAAGACTCAGCCAAC
Downstream primer	Antisense	GCTTGTTCCACGAGTCCCAC

Rat F11R		
Upstream primer	Sense	TCAGACTGCCGTCCAGGTTCC
Downstream primer	Antisense	CTGAAGGTGATGCCACTGGATGAG

**Table 3:** List of biological processes and KEGG pathways that are significantly related to the shared genes.

Category	Term	Count	*p* value
Biology process	GO: 0019882—antigen processing and presentation	14	5.80*E* − 09
	GO: 0006955—immune response	27	1.10*E* − 07
	GO: 0010033—response to organic substance	42	4.04*E* − 07
	GO: 0006631—fatty acid metabolic process	17	6.90*E* − 07
	GO: 0009725—response to hormone stimulus	26	1.70*E* − 05
	GO: 0009719—response to endogenous stimulus	28	1.56*E* − 05
	GO: 0006270—DNA replication initiation	5	2.58*E* − 05
	GO: 0006952—defense response	22	2.99*E* − 05
	GO: 0009611—response to wounding	22	7.18*E* − 05
	GO: 0008610—lipid biosynthetic process	17	1.09*E* − 04
	GO: 0042493—response to drug	18	2.01*E* − 04
	GO: 0014070—response to organic cyclic substance	14	2.25*E* − 04
	GO: 0055114—oxidation reduction	26	3.12*E* − 04

KEGG pathway	rno04612: antigen processing and presentation^*∗*^	12	6.14*E* − 06
	rno04514: cell adhesion molecules (CAMs)^*∗*^	15	9.14*E* − 06
	rno00830: retinol metabolism^*∗*^	8	4.48*E* − 04
	rno03030: DNA replication	6	0.001293
	rno04670: leukocyte transendothelial migration^*∗*^	10	0.001554
	rno00900: terpenoid backbone biosynthesis	4	0.003955
	rno03320: PPAR signaling pathway^*∗*^	7	0.006543
	rno00071: fatty acid metabolism^*∗*^	5	0.017044
	rno04110: cell cycle	8	0.029938

^*∗*^Overlapping with the cholestasis-related pathway in CTD.

## Data Availability

The data used to support the findings of this study are available from the corresponding author upon request.

## Abbreviations

SHCZF: San-Huang-Chai-Zhu formula
ANTI: Alpha-naphthylisothiocyanate
ULN: Upper limit of normal
PSC: Primary sclerosing cholangitis
PBC: Primary biliary cholangitis
SAMe: S-Adenosylmethionine
UDCA: Ursodeoxycholic acid
FDA: Food and Drug Administration
ADR: Adverse drug reaction
FXR: Farnesoid *X* receptor
PXR: Pregnane *X* receptor
PPAR: Peroxisome proliferator-activated receptor
SHP: Small heterodimer partner
TGR5: G-protein coupled receptor 5
DDC: 3,5-Diethoxycarbonyl-1,4-dihydrocollidine
AIC: Acute intrahepatic cholestasis
TCM: Traditional Chinese medicine
HPLC: High-performance liquid chromatography
WGCNA: Weighted gene coexpression network analysis
STEM: Short time-series expression miner
CTD: Comparative Toxicogenomics Database
CAMs: Cell adhesion molecules
DBI: Diazepam binding inhibitor
ACBP: Acetyl-CoA binding protein
HACL1: 2-Hydroxyacyl-CoA lyase
JAM-A: Junctional adhesion molecule A
MC: Microscopic colitis.
